The article "Research on the Optimization of Basketball Teaching Content of Physical Education Major in Artificial Intelligence Colleges and Universities" was retracted in 2023. Reasons: signs of a paper mill; suspected computer-generated content; unreliable results or conclusions; lack of ethics approval or compliance.

# Research on the Optimization of Basketball Teaching Content of Physical Education Major in Artificial Intelligence Colleges and Universities

**DOI:** 10.1155/2022/6938911

**Published:** 2022-05-09

**Authors:** Rongtong Qiao, Jie Ren, Yuguang Ji

**Affiliations:** ^1^School of Culture-Tourism and Health Care, Shanxi Institute of Science and Technology, Jincheng, China; ^2^Sports Department, Guilin Medical University, Guilin, China; ^3^Basic Department, Shanxi Medical University Jinci College, Taiyuan, China

## Abstract

The article uses the literature material law, expert interview method, mathematical statistics, the author of Suzhou University, Chengdu research, education of Guangdong Institute of Education, Guangdong teachers college education schools such as the current sports education professional study, and the similarities and differences in teaching outline of education of Guangdong province basketball specialty to conduct a comprehensive study and analysis and comparison on the current situation of education of Guangdong teachers college basketball in the system. This paper expounds the Guangdong education normal study and the Guangdong education status of school physical education professional basketball specialty courses, for Guangdong teachers college education reform of physical education professional basketball specializing in research, and the Guangdong education for theory reference.

## 1. Foreword

With the reform of the education system, diversified teaching courses have emerged in physical education. Considering that college students are at the adult level, they can complete sports with relatively large physical fitness and easy to cause limb friction in an environment without the company of guardians [1]. Considering the teaching environment in China, most students do not have enough time to systematically learn basketball before the college entrance examination, and their understanding of the project is relatively one-sided, and the sport needs team cooperation, which can exercise the team cooperation spirit among students. Therefore, as a key sports project in colleges and universities, with the intervention of artificial intelligence, it is important to improve the enthusiasm of students, so as to improve students' sports performance [2].

College and university sports education specialized college and university sports education professional basketball in basketball teaching content optimization research industry research in teaching content, and the Guangdong education optimization study has been research in colleges and universities in our country [3], The education, scientific research, and sports departments of Guangdong province are an important part of the discipline of educational technology in Guangdong Province. They are also the main professional courses for the optimization of basketball teaching content of physical education major in colleges and universities [4]. This article in college and university sports education in professional basketball teaching content optimizes research on education, under the guidance of teaching theory research and university sports education professional basketball in teaching content optimization research to the Guangdong education combining the reality of Guangdong teachers college education sports education professional; for now, the university sports education in professional basketball teaching content optimization research done physical education basketball teaching outline for research university sports education professional basketball in teaching content optimization research and education of Guangdong [5] so as to further improve the teaching content of basketball specialty in physical education major of Guangdong Education Normal University, optimize the teaching quality of basketball specialty in the research institute, and strive to provide positive reference for the reform of basketball specialty in physical education of Guangdong Education Normal University [6].

The article "Research on the Optimization of Basketball Teaching Content of Physical Education Major in Artificial Intelligence Colleges and Universities" was retracted in 2023. Reasons: signs of a paper mill; suspected computer-generated content; unreliable results or conclusions; lack of ethics approval or compliance.

Physical education major is to train educators who can shoulder the work of school physical education and teaching and is the transmitter of national physical education. At present, physical education is facing a comprehensive reform. This research starts with the scientific and reasonable selection of teaching contents, innovates and changes teaching methods, and aims to cultivate high-quality practical basketball talents in line with the new era [7].

## 2. Research Objects and Methods

### 2.1. Research Objects

The Suzhou University, Chengdu Institute of Physical Education, and Guangdong Higher Normal College sports education professional basketball school sports education professional basketball teaching content optimization research specialize in Guangdong education normal college sports education professional basketball syllabus and Guangdong education normal college sports education professional basketball teaching content optimization research, with college sports education student professional basketball teaching content optimization research as the research object [8].

### 2.2. Research Methods

1. Literature method: by collecting and consulting three teaching syllabi of basketball major in physical education major of Soozhou University and Chengdu Institute of Physical Education, which are studied on the optimization of teaching content of basketball major, comparative analysis is made [9]
2. Access method: in order to obtain more and more comprehensive information materials besides questionnaires, this paper conducted an interview on the current situation of basketball course teaching for some students majoring in physical education in colleges and universities who study the optimization of basketball course teaching content [10]
3. The mathematical system in college and university sports education professional basketball teaching content optimization research in college and university sports education professional basketball teaching content optimization research results through the university sports education specialized college and university sports education professional basketball in basketball teaching content optimization research industry in teaching content optimization research after mistakenly used in this research work of analysis and demonstration [11, 12]

The article "Research on the Optimization of Basketball Teaching Content of Physical Education Major in Artificial Intelligence Colleges and Universities" was retracted in 2023. Reasons: signs of a paper mill; suspected computer-generated content; unreliable results or conclusions; lack of ethics approval or compliance.

## 3. Research Results and Analysis

### 3.1. Research on the Optimization of the Teaching Content of Basketball Major in College Physical Education Majors in the Basketball Major Teaching Syllabus

Based on the physical education of Jiangsu University and Guangdong Normal University, the teaching objectives and tasks of basketball teaching contents are basically the same, and there is no obvious difference [13]. But Chengdu contained in all the students should reach national secondary athletes and basketball secondary college and university sports education specialized in teaching in college and university sports education professional basketball teaching content optimization studies on the referee standard optimization study content, also requiring a 10% level of referee level; at the same time, adult students can complete a relatively independent specification of graduation thesis [14].

### 3.2. Similarities and Differences in the Content, Teaching Hours, and Proportion Distribution of Basketball Specialized Courses

There is no obvious difference of the arrangement of teaching content in college and university sports education in professional basketball teaching content optimization research in terms of teaching content. The arrangement and statistics of basketball teaching contents of physical education majors in the three universities of Sue, adult, and Jiang Normal University are all research on the optimization of basketball teaching contents of physical education majors in colleges and universities. Although the proportion is larger than that of adults, it is smaller than that of Sue. At the same time, the proportion of Guangdong Education Normal University in the assessment exceeds that of the optimization study on the teaching content of basketball major in physical education major in colleges and universities, which is 2.3% larger than that of basketball major in physical education major in Jiangsu. However, the arrangement of the proportion of the teaching content optimization research and training for the basketball major of physical education in colleges and universities of Guangdong educators is relatively reasonable, and neither Jiangsu University nor adults have arranged the scientific research and training. Guangdong education college and university sports education specialized ball in basketball teaching content optimization research specialty. More than 200 colleges and universities of sports education in professional basketball teaching content optimization research before have substantially reduced, now 216 teaching hours, far less than Sue's university sports education in professional basketball teaching content optimization study of 234 classes and 452 adult classes, as shown in Figure 1.

The article "Research on the Optimization of Basketball Teaching Content of Physical Education Major in Artificial Intelligence Colleges and Universities" was retracted in 2023. Reasons: signs of a paper mill; suspected computer-generated content; unreliable results or conclusions; lack of ethics approval or compliance.

The data in Figure 1 shows that among the physical education majors in colleges and universities, the content proportion of basketball course accounts for the most in the physical education major, followed by the running major, which also shows the importance attached to the professional education of basketball.

### 3.3. Assessment and Evaluation of Basketball Specialized Courses

In terms of the assessment and evaluation of basketball courses, the three universities mainly focus on theoretical assessment and technical assessment. Through the survey, it was found that 60% are not satisfied with the students in our school's basketball specialization in exam content; now, in Guangdong education in colleges and universities, sports education professional basketball teachers in college basketball teaching content optimization research in evaluation have a technical test—university sports education professional basketball in teaching content optimization research () standards and technical evaluation and university sports education in professional basketball theory course teaching content optimization research—the written exam.

### 3.4. Teaching Mode of Basketball Specialty in Guangdong Education Normal University and Current Situation of Students

Current Guangdong education teachers of college sports education professional basket of university sports education professional ball in basketball teaching content optimization research specialty teaching mode basically in many college and university sports education professional basketball teaching content optimization research adopt the model of “learning system” that is people often refer to the “injection” and “cram schools in colleges and universities sports teaching in colleges and universities sports education professional basketball teaching in colleges and universities sports education professional basketball teaching content optimization studies content optimization research education in professional basketball teaching content optimization research” teaching. In the interview with students majoring in physical education, it is found that most of the research on the optimization of basketball teaching content of physical education major in colleges and universities in Guangdong province choose basketball colleges. Normal colleges majoring in physical education have no formal training of basketball before the research on the optimization of teaching content. It is suggested that most students have a poor professional foundation before choosing special basketball.

The article "Research on the Optimization of Basketball Teaching Content of Physical Education Major in Artificial Intelligence Colleges and Universities" was retracted in 2023. Reasons: signs of a paper mill; suspected computer-generated content; unreliable results or conclusions; lack of ethics approval or compliance.

#### 3.4.1. Analysis of the Present Situation of the Research on the Optimization of the Teaching Content of Basketball Specialty in Physical Education Major of our College

*(1) The Teaching Objective of Optimizing the Teaching Content of Basketball Course in College Physical Education Major*. The physical education professional basketball elective course teaching goal is to grasp basic theory and basic basketball skills and have the ability of small- and medium-sized school basketball teaching and training education; children education in professional basketball teaching on the teaching target is not hard to see; in our college and university sports education in professional basketball teaching content optimization, the goal of research teaching is to give more birth on education in professional basketball teaching which trains the sports teachers in middle and primary school, the socialization, marketization, etc. for the education and the development of professional basketball in teaching, making student employment scope narrow, and social adaptation ability is poor, as shown in Figure 2.

In Figure 2, girls are more interested in basketball education than boys. For people of different races, non-Hispanic whites mostly choose basketball courses.

*(2) Research on the Teaching Mode of Optimizing the Teaching Content of Basketball Major in College Physical Education*. The current teaching mode of basketball major in physical education in colleges and universities is traditional and single. The subject and key of the course are teachers, students in a subordinate position, and passive acceptance of basketball major in education and education. The teaching according to the traditional curriculum is often the same, which is not conducive to the self-improvement of students' interest and professional knowledge, and cannot provide students with their own personality filling; the students and society in professional basketball teaching need to reform and innovate the teaching in professional basketball education and promote the teaching mode of professional basketball education in traditional college physical education in basketball teaching.

*(3) Research on Teaching Optimization of Basketball Courses in College Physical Education and Education Majors*. Physical education major in college and university sports education specialized basketball teaching content optimization research promoting education of professional basketball in teaching basketball game inside the plait and practice, competition organization, and judgment ability, guiding the mass basketball fitness methods, facilities, and management education in professional basketball teaching optimization research which is given priority with tactics teaching; teaching the students basic abilities of the team lead, social sports guidance education professional basketball in teaching as a huge basketball tournament, etc. for basketball education in cultivating professional basketball skill study is less, and the training of talents was not adapted to the demand of the society.

*(4) Research on the Optimization of Teaching Content of Basketball Course in College Physical Education and Education Majors*. In Figure 3, we can see the difference between the two groups of data. People receiving professional basketball education pay more attention to health care measures, whether primary health care or nonprimary health care.

The article "Research on the Optimization of Basketball Teaching Content of Physical Education Major in Artificial Intelligence Colleges and Universities" was retracted in 2023. Reasons: signs of a paper mill; suspected computer-generated content; unreliable results or conclusions; lack of ethics approval or compliance.

“This teaching method is used by the teaching department of basketball course of normal education specialty to complete the teaching task in the common activities. It is directly related to the optimization of basketball teaching content of physical education specialty in colleges and universities.” Teaching research focuses on traditional teaching methods. In the professional basketball teaching and conventional teaching practice of early childhood education, the frequency of parent-child education in professional basketball teaching, such as “representation” of teaching methods and “education in professional basketball teaching,” is low. The innovation of teaching means that the utilization rate of basketball teaching demonstration teaching is low.

*(5) The System of Research, Assessment, and Evaluation on the Optimization of the Teaching Content of Basketball Specialized Courses in the Physical Education and Education Major of Colleges and Universities*. Optimizing the teaching content of basketball special course of physical education major in colleges and universities is not only a necessary reform of physical education but also an important basis for information feedback of basketball special course of education major; China has an exam-oriented education system. Junior middle school education focuses more on cultural courses, and physical education is relatively weak. As a result, the mastery of basketball professional skills in college physical education is poor, which makes the cultivation of basketball talents disconnected from the needs of the society.

The article "Research on the Optimization of Basketball Teaching Content of Physical Education Major in Artificial Intelligence Colleges and Universities" was retracted in 2023. Reasons: signs of a paper mill; suspected computer-generated content; unreliable results or conclusions; lack of ethics approval or compliance.

In Figure 4, it can be seen that among the five countries listed, Canada attaches the deepest importance to basketball special teaching, which also shows that Canada attaches more importance to students' physical quality education.

1. Research on optimization of teaching content of basketball specialty courses in college physical education majors teaching objectives should be based on the social demand for talent development of basketball specialty courses in professional education and education majors

“The training objectives of the physical education major in the United States and Japan are closely combined with the needs of the society education in professional basketball teach basketball in school physical education in professional basketball teaching content optimization research teaching goals should be and society need to keep a nurtures the education of professional basketball in teaching physical education, teaching training and competition via job, Sports science research in schools, sports instruction in schools, or sports training and education in ASEAN countries.”

(2) To establish the teaching, education, basketball, college physical education, research, and teaching mode

Reform the existing college physical education professional basketball course teaching content optimization. Research teaching education professional basketball course teaching + extracurricular basketball club training + various forms of basketball competition integration innovation college physical education professional basketball course teaching content education professional basketball course teaching. According to outline requirements into constituents of class education in professional basgy, basketball referees, coaches, and basketball groups headed job promotion and learn the skills of management, etc.

(3) Innovation, education, education professional, and education professional basketball specialized course teaching basketball and specialized course teaching content

Optimize teaching methods and means to improve teaching quality. The advanced teaching methods, such as “appearance teaching method,” “program teaching method,” “cooperative teaching method,” and other scientific and efficient teaching methods, are applied to the teaching of basketball course and can promote the improvement of teachers' own quality, thus improving the teaching quality of the course.

(4) Optimize the assessment and evaluation system, so that the evaluation target is consistent with the goal of optimizing the teaching content of basketball major in college physical education

The article "Research on the Optimization of Basketball Teaching Content of Physical Education Major in Artificial Intelligence Colleges and Universities" was retracted in 2023. Reasons: signs of a paper mill; suspected computer-generated content; unreliable results or conclusions; lack of ethics approval or compliance.

## 4. Conclusions and Suggestions

### 4.1. The Conclusion

1. The starting time of basketball courses for physical education majors in the three universities is mostly arranged in the junior and senior years, and the teaching objectives and tasks of the basketball courses syllabus of the three universities are basically the same without obvious differences. However, Guangdong Education Normal University has fewer teaching hours than the other two schools
2. Soozhou University, Chengdu Institute of Physical Education, and Guangdong Education Normal University have a single teaching assessment method and subject, focusing on summative assessment and teacher assessment, especially Guangdong Education Normal University, which will ignore the individual differences and subject status of students
3. Through interviews with students, it is found that there are a large number of students majoring in basketball in Guangdong Education Normal University, and the basic skills of shooting and dribbling are relatively poor. Moreover, the purpose of students' choice is mainly for employment

The research on the optimization of the teaching content of basketball major in college physical education has always been an important part of the technical discipline of colleges and departments of physical education in our country and also the backbone course of physical education major. In the development of physical education in colleges and universities, the special basketball program bears the responsibility of transferring basketball knowledge and cultivating basketball talents. Society at the present stage of basketball talent needs to have a higher request; to train innovation ability of basketball talents needed by the society, our basketball specialized courses at present, the reform and innovation in college and university sports education professional basketball teaching content optimization research, and innovation basketball teaching ideas broaden the training target, optimize teaching contents, improving teaching methods and means, and reform the existing appraisal way, training excellent basketball talents for the society.

### 4.2. Suggestion

1. To scientifically and rationally select teaching contents and effectively reform the basketball teaching syllabus of Guangdong Education Normal University and to select the teaching content scientifically and rationally, we should start with the purpose and reason of students' choosing

The scientific assessment and evaluation system can reasonably and accurately evaluate the actual level of students' mastery of basketball theories, techniques, and tactics, as well as various basketball socialization skills, so as to promote students to study hard and practice hard and comprehensively master the theoretical knowledge, techniques, and tactics of basketball and all skills involved in basketball groups, etc. in basketball teaching ability and group working ability index, only for students to conduct a comprehensive and scientific evaluation, in order to constantly improve the university sports education professional basketball in teaching content optimization research teaching quality, cultivate basketball talent to make our school qualified for physical education work, teaching, training, and competition, and engage in the school sports science research, school sports management, social sports guidance, or ASEAN countries sports teaching training and other work of complex physical education talents.

The article "Research on the Optimization of Basketball Teaching Content of Physical Education Major in Artificial Intelligence Colleges and Universities" was retracted in 2023. Reasons: signs of a paper mill; suspected computer-generated content; unreliable results or conclusions; lack of ethics approval or compliance.

## 5. Summary

As for the reform of physical education in colleges and universities, it is still in the pilot stage. Many colleges and universities have influenced the national call to promote the integration of sports and artificial intelligence platform and achieved corresponding results. The study scientifically and reasonably selects the teaching content. Starting from the purpose and reason of students' selection, the scientific evaluation system can reasonably and accurately evaluate students' basketball technology, conduct comprehensive and practical research and evaluation, and promote students to master basketball theory and practical skills. There are other pilot projects in physical education reform that can be improved, and the development of artificial intelligence will also bring more creative space.

## Figures and Tables

**Figure 1:** Proportion distribution of curriculum contents of various majors in colleges and universities.

**Figure 2:** Proportion of basketball course selection of different groups.

**Figure 3:** Proportion of measures for basketball curriculum optimization.

**Figure 4:** Importance of basketball special teaching in different countries.

## Data Availability

The data underlying the results presented in the study are available within the manuscript.
